# The Application Value of MRI T2^∗^WI Radiomics Nomogram in Discriminating Hepatocellular Carcinoma from Intrahepatic Cholangiocarcinoma

**DOI:** 10.1155/2022/7099476

**Published:** 2022-09-27

**Authors:** Feng Huang, Xiaoyun Liu, Peng Liu, Dan Xu, Zeda Li, Huashan Lin, An Xie

**Affiliations:** ^1^Department of Radiology, Hunan Provincial People's Hospital (The First Affiliated Hospital of Hunan Normal University), Changsha 410005, China; ^2^Department of Pharmaceutical Diagnosis, GE Healthcare, Changsha 410005, China

## Abstract

**Objective:**

To establish and validate an MRI T2^∗^WI-based radiomics nomogram model and to discriminate hepatocellular carcinoma (HCC) from intrahepatic cholangiocarcinoma (ICCA).

**Methods:**

174 patients were retrospectively collected, who were diagnosed with primary hepatic carcinoma by surgery or puncture pathology and received preoperative MRI scans including T2^∗^WI scans. There were 113 cases of HCC and 61 cases of mass-type ICCA. T2^∗^WI was used for feature extraction, the extent of the lesions was manually outlined at the largest lesions layer of the T2^∗^WI, and the feature dimension reduction was performed by the mRMR and LASSO to obtain the optimal feature set. The radiomics features and clinical risk factors were combined to establish the radiomics nomogram model. In both training and validation groups, calibration curves and ROC curves were applied to validate the efficacy of the established model. Finally, calibration curves were applied to assess the degree of fitting and DCA to assess the clinical utility of the established model.

**Results:**

The radiomics model had the AUC of 0.90 (95% CI, 0.85–0.96) and 0.91 (95% CI, 0.83–0.99) in the training and validation groups, respectively; the AUC of the radiomics nomogram was 0.97 (95% CI, 0.94–0.99) in the training group and 0.95 (95% CI, 0.95–0.99) in the validation group. DCA suggested the clinical application value of the nomogram model.

**Conclusion:**

Radiomics nomogram model based on MRI T2^∗^WI scan without enhancement can be used to discriminate HCC from ICCA.

## 1. Introduction

Primary hepatic carcinoma ranked first among the malignant tumor of the liver in China. It can be classified into hepatocellular carcinoma (HCC), intrahepatic cholangiocarcinoma (ICCA), and mixed type of hepatocarcinoma. HCC has the second-highest mortality among tumors in China [1], and ICCA, a subtype of cholangiocarcinoma, is second only to HCC, accounting for 5%–10% of primary hepatic carcinoma [2]. Different types of primary hepatic carcinoma vary greatly in prognosis and responses to adjuvant therapies. Their symptoms, serum tumor markers, and imaging manifestations have differences as well as similarities. Although it has been reported that radiologic diagnostic models based on CT and MRI images can rapidly differentiate HCC from ICCA [3, 4], especially noncontrast MRI which is difficult for radiologists to correctly distinguish them accordingly, so far, there is no relevant literature report on noncontrast MRI based on T2^∗^WI to differentiate ICCA from HCC. Therefore, it would be of great benefit to both doctors and patients to discover a method to identify different types of primary hepatic carcinoma on non-contrast-enhanced MRI scans.

MRI, with multiparametric and arbitrary layer imaging, has become one of the routine examinations for occupying liver lesions. T2^∗^WI is a novel noninvasive functional imaging technique. It can obtain magnetic sensitivity variability between tissues and thus is used to evaluate the biological properties of tumor tissue [5]. Radiomics make it possible to extract enormous image features and transform them into data that can quantitatively characterize tumor biology. A great deal of clinical data can be integrated to develop models in favor of clinical decision-making and tumor heterogeneity quantification, which enables noninvasive, comprehensive, and dynamic accurate treatment and prognosis prediction of diseases [6–8]. Comprehensive analysis of multiple features tends to be the greatest encouraging approach. Nomograms can parallelly study multiple features and transform complex regression equations into visualized tables that present the quantitative assignment of different predictors, which can be helpful for clinic treatment [9–11]. This research attempts to develop and validate the radiomics nomogram model based on MRI T2^∗^WI sequences and clinical risk factors, and it is aimed at comparing its ability to discriminate HCC from ICCA.

## 2. Materials and Methods

### 2.1. Patients

Patients who were hospitalized in Hunan Provincial People's Hospital from October 2019 to December 2021 were retrospectively included. Inclusion criteria were as follows: (1) patients with HCC or ICCA confirmed pathologically by surgery or puncture biopsy; (2) MRI scans were performed 3 weeks before surgery or puncture biopsy; (3) all patients underwent a preoperative MRI scans including T2^∗^WI sequence on the same MRI device; (4) patients who did not receive tumor-related treatment before the examination; and (5) the maximum diameter of the lesion was ≥10 mm. Exclusion criteria were as follows: (1) MR image quality could not meet the diagnostic requirements; (2) clinical information was incomplete; and (3) patients had existing intrahepatic or distant metastases. Finally, 174 patients were included in the study. 113 patients with HCC consisted of 102 males and 11 females, aged 29–80 years, with a mean age of 54.9 ± 11.4 years. 61 patients with ICCA consisted of 36 males and 25 females, aged 29–84 years, with a mean age of 58.4 ± 10.4 years. According to the ratio of 7 : 3, all cases were randomly assigned, with 123 and 51 cases in the training and validation group, respectively. The flowchart for the screening of patients is presented in Figure 1.

### 2.2. MRI Image Acquisition

All images were obtained by a Philips Ingenia DNA 3.0 T MR scanner with a 32-channel phased-array coil. The liver MRI scan and mDixon-Quant quantitative imaging were performed. mDixon-Quant generated T2^∗^WI. mDixon-Quant used breath-hold 3D volume interpolated spoiled gradient recalled echo sequence, with a TR of 9.1 ms, a TE of 1.33 ms, an echo spacing of 1.3 ms, the layer thickness of 5 mm, an interval of 0 mm, a FOV of 400 mm × 350mm, and a matrix of 224 × 170.

### 2.3. Image Segmentation and Radiomics Feature Extraction

T2^∗^WI were selected with the largest lesion layer in DICOM format and imported into the open-source ITK-SNAP software (version 3.8.0). The lesion extent was manually segmented by 2 physicians with 10 years of experience in diagnostic abdominal MRI (Figures 2(a)–2(d)). Thirty-two liver lesions were selected randomly to compute intraobserver and interobserver consistency on feature extraction. Two weeks later, a physician unaware of the results of tumor pathology extracted radiomics features using the same method and calculated the intraclass correlation coefficient (ICC) to assess the reproducibility of radiomics feature extraction. ICC > 0.80 indicated good consistency, and only features with ICC > 0.8 were included in feature screening and modeling. AK (Artificial Kit, GE Healthcare) software was used to extract features.

### 2.4. Development of Radiomics Features

Max-relevance and min-redundancy (mRMR) algorithms were used to remove redundant and irrelevant features from the radiomics features extracted from the T2^∗^WI and retain the 20 most meaningful features. Then, the least absolute shrinkage and selection operator algorithm (LASSO) was used to further reduce the dimensionality of the 20 features to obtain the optimal feature set [12]. The linear combination of selected features was used to calculate the radiomics score for discriminating HCC from ICCA by weighting their respective coefficients. The receiver operating characteristic (ROC) curves were performed to evaluate the discriminative efficacy of the radiomics features of the two sets.

### 2.5. Development of Radiomics Nomogram

Clinical risk factors included gender, age, hepatitis B virus (HBV), alpha-fetoprotein (AFP), carcinoma embryonic antigen (CEA), and carbohydrate antigen 199 (CA199). Univariate and multivariate logistic regression was performed to select risk factors, and nomograms were established based on multivariate regression in the training group.

### 2.6. Validation and Performance Evaluation of Radiomics Nomogram

The predictive efficacy of radiomics nomogram in the training group was evaluated using the ROC curve, and the consistency between the observed and predicted results was evaluated by the calibration curve. Classification of primary hepatic carcinoma cases was in good consistency with the prediction accuracy based on radiomics nomogram when the calibration curve got close to the diagonal line. The Hosmer-Lemeshow test was performed to identify the degree of fitting of radiomics nomogram. Both the training and validation groups used the same method to validate the radiomics nomogram.

Decision curve analysis (DCA) was used to assess the clinical utility of radiomics nomogram in the validation group. ROC curve was used to calculate the area under curve (AUC), and this only considers the specificity and sensitivity of the method, while DCA quantifies the net benefits at different risk thresholds in the validation group and determines the clinical benefits of radiomics nomogram [13].

### 2.7. Statistical Analysis

R language (version 4.1.0) software was used to perform statistical analysis. Continuous variables were presented by median ± range interquartile. Quantitative data were compared by independent sample *t*-test or *U*-test. Categorical variables were presented by numbers and percentages and compared by the *χ*^2^ test; ROC curve, calibration curve, and DCA were performed to assess the discrimination efficiency of the radiomics nomogram. A two-sided *P* < 0.05 was considered that the differences were statistically significant.

## 3. Results

### 3.1. Patient Characteristics

There were 123 cases in the training group, including 80 cases of HCC and 43 cases of ICCA. There were 51 cases in the validation group, including 33 cases of HCC and 18 cases of ICCA. No significant difference was shown in the age of onset, gender, HBV, AFP, CEA, and CA199 between the cases in the training and validation groups (*P* > 0.05). This proved the reasonableness of the case assignment between the training and validation groups. There were statistically significant differences between HCC and ICCA in terms of gender, HBV, AFP, and CEA within the training and validation groups (*P* < 0.05), as detailed in Table 1. The proportion of males between HCC and ICCA showed a statistical difference (90.3% vs. 59%, *P* < 0.0001). AFP positivity rate was 60.2% in HCC and 26.2% in ICCA, with statistically significant difference (*P* < 0.0001). Only 1 of 113 HCC patients was CEA positive, and the positive rate of ICCA was 32.8%, which was statistically significant (*P* < 0.0001). The results of univariate logistic regression of HCC and ICCA are shown in Table 2.

### 3.2. Radiomics Feature Screening, Model Development, and Validation

Among the 932 total features, 861 had ICC > 0.8, accounting for 92.4%, with good intra- and interobserver consistency. The optimized model was calculated by the LASSO regression algorithm and the tenfold cross-validation method with the parameter *λ* of 0.0005 (Figure 3(a)). Eight first-order statistic features, 3 gray-level size zone matrix (GLSZM), 4 gray-level cooccurrence matrix (GLCM), and 1 gray-level run-length matrix (GLRLM) were screened, with a total of 16 nonzero coefficients of the features (Figure 3(b)). The weighting coefficients of each feature are shown in Figure 3(c). A significant difference was shown between the radiomics scores of HCC and ICCA in the training and validation groups (*P* < 0.001, Figure 3(d)). Radiomics model had AUCs of 0.90 (95% CI, 0.85–0.96) and 0.91 (95% CI, 0.83–0.99) in the training and validation groups, respectively (Figures 4(a) and 4(b)).

### 3.3. Development and Validation of the Radiomics Nomogram Model

The results of the multivariate logistic regression of the clinicopathological influence factors on the discrimination of HCC and ICCA are shown in Table 2. The nomogram model included radiomics features and clinical risk factors (Figure 5(a)). Radiomics nomogram exhibited an AUC of 0.97 (95% CI, 0.94–0.99) in the training group and 0.95 (95% CI, 0.91–1.00) in the validation group (Figures 4(a) and 4(b)). Figures 5(b) and 5(c) present the calibration curves. The diagonal line is the ideal model curve, the red line is the actual prediction of the model, and the better fit of the red line to the diagonal line represents the better fit of the model to the actual situation. The accuracy, sensitivity, and specificity of the different discriminative prediction models are shown in Table 3. Calibration curves using the Hosmer-Lemeshow test displayed good consistency between the true classification of HCC and ICCA and the prediction probabilities based on the radiomics nomogram model (*P* = 0.983). DCA showed a high net benefit of the model in the threshold range of 0.1–1.0 (Figure 5(d)).

## 4. Discussion

The surgical methods and prognosis of primary hepatic carcinoma are completely different for different pathological types [14]. Kianmanesh et al. [15] reported a 5-year survival rate of 50% after surgical resection for HCC compared to 39% after radical resection for ICCA [16]. Currently, the main examination methods to discriminate between HCC and ICCA are CT and MRI [14]. However, both methods are subjective to the observer and still produce many misdiagnoses for HCC and ICCA that are smaller in size or have atypical enhancement; especially, the diagnostic accuracy is even lower when contrast enhancement is not performed. Literature has reported that the misdiagnosis rate can reach 50% in discriminating intrahepatic tumor types based only on preoperative CT versus MRI [17]. Therefore, methods with higher diagnostic efficacy need to be explored. The general data of the present study showed a significantly higher incidence of HCC in males than in females, which was consistent with the study of Pinheiro et al. [18] and might be related to the following genetic aspects: the higher incidence of hepatitis B infection in males, the gender specificity of estrogen and its receptors with HCC [19], and the higher adiponectin in females compared to males, which show anti-HCC effect [20]. Besides, alcohol abuse and social stress in males are also associated. When pregnancy, active liver disease, and gastrointestinal tumors are excluded, AFP ≥ 400 *μ*g/l is highly suggestive of HCC [21]. The AFP positivity rate in this study was 60.2% for HCC and 26.2% for ICCA (*P* < 0.0001), and the odds ratio (OR) and 95% CI for AFP and CEA positivity were 0.2449 and 46.815, respectively (*P* < 0.006 and 0.002). Although these tumor serum markers were statistically different, the specificity was not high [21]. The AUC for discriminating HCC with ICCA using clinical features was only 0.88 (95% CI, 0.81–0.95) in the training group and 0.83 (95% CI, 0.72–0.94) in the validation group.

The sequence of a multiecho gradient recalled echo (GRE) T2^∗^WI is a relatively new MRI technique. It can detect the smallest changes in uniformity in the magnetic field and can improve the rate of small lesion detection. In addition, the T2^∗^ value can indirectly reflect changes in tissue biochemical components, such as iron deposits and microbleeds. Moreover, it can be used for the early diagnosis and quantitative diagnosis of some diseases [22]. HCC cells were arranged in strips separated by blood sinuses with less fibrous interstitium [14], whereas ICCA was predominantly adenocarcinoma originating from the lining epithelium of the intrahepatic bile duct and its branches to the interlobular fine bile duct tree, with cuboidal or columnar cancer cells and abundant fibrous tissue around the cancer cells, often accompanied by a dilatation of the fine bile ducts [2]. Compared to HCC, the large amount of sparse fibrous interstitium and dilated interlobular fine bile ducts in the center of ICCA promote the diffusive movement of water molecules [23–25]. This results in less random fluctuations in the interproton surrounding the magnetic environment and slower proton out of phase, prolonging the tissue T2^∗^ values. Figures 2(C1) and 2(C2) show that the ICCA signal is significantly higher than that of HCC on T2^∗^WI.

Sun et al. [26] reported that magnetic resonance blood oxygen level parameters R2^∗^ and T2^∗^ and their associated measurements were correlated with the clinical and pathological features of HCC. Zhang et al. [27] investigated the significance of mean platelet volume (MPV) in discriminating HCC from ICCA and found that MPV correlation discrimination had the AUC, sensitivity, and specificity of 0.698, 80.2%, and 54.1%, respectively. After the combination of sex, AFP, CA19-9, HBsAg, and MPV, the diagnostic efficiency was improved, with an AUC of 0.907, a sensitivity of 85.4%, and a specificity of 82%. The study of Zhang et al. demonstrated that the combination of biomarkers based on MPV was sufficiently accurate in differentiating HCC from ICCA. This study proposed T2^∗^WI radiomics nomogram based on MRI plain scan and showed an AUC of 0.95, sensitivity of 81%, and specificity of 96.7% in the validation group, which exhibited better performance than the utility of mean platelet volume. The radiomics and clinical features used in the study can be acquired in a noninvasive approach before surgery, thus demonstrating good utility.

The discrimination and calibration performance of the radiomics nomogram is not representative of the clinical application value, and DCA can effectively assess the ability of the model to discriminate HCC from ICCA in clinical work. In the threshold range of 0.1–1.0, radiomics nomogram offers more net benefit than all diagnostic results for HCC or ICCA.

Based on the MRI T2^∗^WI radiomics features and clinical features, this study comprehensively considered the clinical features and imaging features of different pathological types of primary hepatic carcinoma and used their respective weights to develop the nomogram model for discriminating HCC from ICCA. The T2^∗^ values of liver tissues are influenced not only by the tissue microenvironment but also by iron deposition, tumor tissue cystic degeneration, hemorrhage, and necrosis. Though there are significant differences in T2^∗^7 values between HCC and ICCA, T2^∗^ values alone may be biased by the choice of observer region of interest (ROI). The use of tissue features extracted by outlining all lesion areas at the largest tumor tissue layer can better reflect the specific differences between HCC and ICCA tissues and help to accurately identify HCC and ICCA.

The present study has some limitations. First, patients came from a single center and the sample size was limited, especially the mixed type of hepatocarcinoma was not included in the study population, and a large sample multicenter study is still needed. Second, due to the low resolution of T2^∗^WI, T2WI are sometimes needed to refer to when outlining the tumor tissue, which however does not affect the results of this study. To comprehensively assess the discriminative ability of HCC and ICCA in the MRI plain scans, more other imaging features can be added in future studies. Third, this study is a retrospective study, and double-blind prospective studies should be used in the future to overcome selective bias.

## 5. Conclusion

The nomogram model based on MRI T2^∗^WI radiomics and clinical risk factors showed good discriminative performance in discriminating HCC from ICCA. This model uses no contrast injection and can better predict the pathological type of primary hepatic carcinoma preoperatively and help clinicians to choose the best treatment plan, which has high clinical application value. MRI T2^∗^WI can be used to differentiate HCC from ICCA when patients have certain contraindications that do not allow enhanced MR.

## Figures and Tables

**Figure 1:** Workflow of the study.

**Figure 2:** A1-D1 and A2-D2 show the imaging of T1WI, T2WI, T2^∗^WI, and ROI segmentation on T2^∗^WI in the case of HCC and ICCA, respectively. T2^∗^ value in HCC and ICCA patient is 30.21 ms and 58.97 ms.

**Figure 3:** LASSO algorithm for radiomics feature selection. (a) Mean square error path using 10-fold cross-validation; (b) LASSO coefficient profiles of the radiomics features. (c) Rad-score was calculated by summing the selected features weighted by their coefficients. (d) 0 HCC and 1 ICC, rad scores from class 0 and class 1 on the training set and validation set, respectively.

**Figure 4:** ROC curves of the radiomics clinics and nomogram in the training and validation sets: (a) training set; (b) validation set.

**Figure 5:** The evaluation of the degree of fitting for the combined model and comparison of clinical utility of three models: (a) radiomics nomogram with radiomics signature and clinical factors; (b) calibration curves of the radiomics nomogram in the training; (c) validation; (d) DCA of the radiomics nomogram.

**Table 1:** Clinical features.

Variable	Training set (*n* = 123)			Validation set (*n* = 51)			Combined		
	HCC (*n* = 80)	ICCA (*n* = 43)	*P*	HCC (*n* = 33)	ICCA (*n* = 18)	*P*	Training	Validation	*P*
Gender (*n* (%))									
Female	8 (10.0)	16 (37.2)		3 (9.1)	9 (50.0)		24 (19.5)	12 (23.5)	
Male	72 (90.0)	27 (62.8)	0.0007	30 (90.0)	9 (50.0)	0.0032	99 (80.5)	39 (76.5)	0.6966
Age (years)									
Mean (SD)	54.1 (12.3)	59.3 (10)	0.0174	56.8 (8.8)	56.4 (11.6)	0.8818	55.9 (11.8)	56.7 (9.8)	0.6990
HBV (*n* (%))									
No	9 (11.2)	12 (27.9)		1 (3.0)	6 (33.3)		21 (17.1)	7 (13.7)	
Yes	71 (88.8)	31 (72.1)	0.0366	32 (97.0)	12 (66.7)	0.0098	102 (82.9)	44 (86.3)	0.7487
AFP (ng/ml)									
<20	31 (38.8)	31 (72.1)		14 (42.4)	14 (77.8)		62 (50.4)	28 (54.9)	
≥20	49 (61.2)	12 (27.9)	0.0008	19 (57.6)	4 (22.2)	0.0331	61 (49.6)	23 (45.1)	0.7088
CEA (ng/ml)									
<5	79 (98.8)	27 (62.8)		33 (100.0)	14 (77.8)		106 (86.2)	47 (92.2)	
≥5	1 (1.2)	16 (37.2)	0.0001	0 (0.0)	4 (22.2)	0.0228	17 (13.8)	4 (7.8)	0.3974
CA199 (U/ml)									
<35	57 (71.2)	24 (55.8)		20 (60.6)	14 (77.8)		81 (65.9)	34 (66.7)	
≥35	23 (28.8)	19 (44.2)	0.1280	13 (39.4)	4 (22.2)	0.3511	42 (34.1)	17 (33.3)	1.0000

Data are feature's numbers or means, with percentage in parentheses.

**Table 2:** Risk factors.

Variable	Univariate logistic regression		Multivariate logistic regression	
	OR (95% CI)	*P*	OR (95% CI)	*P*
Gender	0.1875 (0.072; 0.4882)	0.0006	0.20 (0.06; 0.64)	0.0072
Age	1.0407 (1.0058; 1.0769)	0.0219	NA	NA
HBV	0.3275 (0.1252; 0.8567)	0.0229	NA	NA
AFP	0.2449 (0.1096; 0.5472)	0.0006	0.15 (0.05-0.46)	0.0008
CEA	46.815 (5.925; 369.876)	0.0002	85.97 (9.13; 809.83)	<0.0001
CA199	1.9619 (0.9062; 4.2477)	0.0873	2.17 (0.79; 5.94)	0.1327

OR: odds ratio; NA: not available.

**Table 3:** Accuracy and predictive value between three models.

Model	Accuracy	95% CI	Sensitivity	Specificity	PPV	NPV	Cutoff
Training							
Radiomics	0.837	0.760-0.898	0.930	0.788	0.702	0.955	NA
Clinics	0.837	0.760-0.898	0.767	0.875	0.767	0.875	NA
Nomogram	0.935	0.876-0.972	0.860	0.975	0.949	0.929	NA
Validation							
Radiomics	0.804	0.668-0.902	0.778	0.818	0.700	0.871	-0.819
Clinics	0.706	0.562-0.825	0.611	0.757	0.579	0.781	-0.345
Nomogram	0.902	0.786-0.967	0.810	0.967	0.944	0.879	-0.900

CI: confidence interval; PPV: positive-predictive value; NPV: negative-predictive value.

## Data Availability

No additional data are available.
